# Influence of the Physical Inclusion of ZrO_2_/TiO_2_ Nanoparticles on Physical, Mechanical, and Morphological Characteristics of PMMA-Based Interim Restorative Material

This article has been retracted.

**DOI:** 10.1155/2022/1743019

**Published:** 2022-08-19

**Authors:** Ali Alrahlah, Rawaiz Khan, Fahim Vohra, Ibrahim M. Alqahtani, Adel A. Alruhaymi, Sajjad Haider, Abdel-Basit Al-Odayni, Waseem Sharaf Saeed, H. C. Ananda Murthy, Leonel S. Bautista

**Affiliations:** ^1^Engineer Abdullah Bugshan Research Chair for Dental and Oral Rehabilitation, College of Dentistry, King Saud University, Riyadh 11545, Saudi Arabia; ^2^Restorative Dental Sciences Department, College of Dentistry, King Saud University, Riyadh 11545, Saudi Arabia; ^3^Department of Prosthetic Dental Science, College of Dentistry, King Saud University, Riyadh 11545, Saudi Arabia; ^4^Public Security Medical Services, Security Patrols Medical Center, Riyadh, Saudi Arabia; ^5^Prince Mohammed bin Naif Medical Center, King Fahad Security College, Riyadh, Saudi Arabia; ^6^Department of Chemical Engineering, College of Engineering, King Saud University, PO Box 800, Riyadh 11421, Saudi Arabia; ^7^Department of Applied Chemistry, School of Applied Natural Science, Adama Science and Technology University, P O Box, 1888 Adama, Ethiopia; ^8^Department of Prosthodontics, Saveetha Dental College & Hospital, Saveetha Institute of Medical and technical science (SIMAT), Saveetha University, -600077, Chennai, Tamil Nadu, India

## Abstract

Polymethyl methacrylate (PMMA) is often used in restorative dentistry for its easy fabrication, aesthetics, and low cost for interim restorations. However, poor mechanical properties to withstand complex masticatory forces are a concern for clinicians. Therefore, this study aimed to modify a commercially available PMMA-based temporary restorative material by adding TiO_2_ and ZrO_2_ nanoparticles in different percentages as fillers and to investigate its physio-mechanical properties. Different percentages (0, 0.5, 1.5, and 3.0 wt%) of TiO_2_ and ZrO_2_ nanoparticles were mixed with the pristine PMMA resin (powder to liquid ratio: 1 : 1) and homogenized using high-speed mixer. The composites obtained were analyzed for their flexural strength (F.S.), elastic modulus (E.M.), Vickers hardness (H.V.), surface roughness Ra, morphology and water contact angle (WCA). The mean average was determined with standard deviation (SD) to analyze the results, and a basic comparison test was conducted. The results inferred that adding a small amount (0.5 wt%) of TiO_2_ and ZrO_2_ nanoparticles (NPs) could significantly enhance the physio-mechanical and morphological characteristics of PMMA interim restorations. EM and surface hardness increased with increasing filler content, with 3.0 wt.% ZrO_2_ exhibiting the highest EM (3851.28 MPa), followed by 3.0 wt.% TiO_2_ (3632.34 MPa). The WCA was significantly reduced from 91.32 ± 4.21° (control) to 66.30 ± 4.23° for 3.0 wt.% ZrO_2_ and 69.88 ± 3.55° for 3.0 wt.% TiO_2_. Therefore, TiO_2_ and ZrO_2_ NPs could potentially be used as fillers to improve the performance of PMMA and similar interim restorations.

## 1. Introduction

In restorative dentistry, temporary restorations are generally adopted amid tooth preparation and placement of the final restoration [1, 2]. Provisional restorations are also beneficial for diagnostic purposes, where the functional, stabilizing, occlusal, and aesthetic parameters are established to determine an optimal therapeutic efficacy before the final prosthesis is completed [3]. Therefore, provisional restorations have acquired immense importance in restorative dentistry due to very demanding aesthetical outputs and early diagnostic of the performance of final restorations. By adopting the provisional restoration approach, the dentists maintain their patients' confidence by implementing this temporary phase of therapy and foresee critical deficiencies in the ultimate restoration prior to installation [4, 5]. Therefore, provisional restorative materials are usually employed to safeguard the prepared teeth until the final rehabilitation.

Temporary restorations are exposed to masticatory forces and need adequate mechanical strength in order to withstand the recurrent functional stresses of the oral environment. The mechanical properties of intermediate restorations play a vital role in helping practitioners decide on the appropriate material to use in specific clinical conditions such as vertical dimensional changes in full oral rehabilitation, temporomandibular joint disorder, and long-span fixed prostheses [4]. To achieve good mechanical strength in the oral environment, the dental material must be reinforced with such nanofillers that provide adequate mechanical strength to the tooth and are also safe to use. Ceramic nanoparticles such as TiO_2_ and ZrO_2_ NPs are primarily used for this purpose [6, 7]. TiO_2_ NPs are white solids and considered technologically crucial due to their various properties [8, 9] such as ease of synthesis, good tensile strength [10, 11] adequate biocompatibility [12], antibacterial activity [13], and photocatalytic activity [11]. TiO_2_ NPs are widely used as catalyst supports in biomedicine, water and air purification [14], pigments [14], cosmetics, solar cells [15], and tissue engineering [16–18]. ZrO_2_ was first introduced in 1789 by Martin Heinrich Klaproth. Since then, it has been used as a pigment for ceramics. It occurs in three crystalline forms at different temperatures. The common one is monoclinic (at normal temperature), while the cubic and tetragonal crystalline forms occurs at elevated temperatures. The toughness of ZrO_2_ increases with decreasing temperature during phase transformation from tetragonal to monoclinic (a stable phase). This property of ZrO_2_ can be used to modify its mechanical properties [18]. Currently, ZrO_2_ is frequently utilized in various dental applications such as dental implants, abutments, crown prostheses, and post-implant restorations [19, 20].

PMMA is a popular polymer material in restorative dentistry, particularly for indirect restorations such as dentures, temporary crowns, and bridges [21–23]. This material is cost-effective, easy to fabricate, and has excellent aesthetical properties. However, its stiffness and fracture toughness are insufficient to withstand the complex masticatory forces [24, 25]. Therefore, the poor mechanical properties limit its clinical application for temporary crowns and fixed bridges for a transitional period [23, 26].

Several efforts have been made to improve the mechanical performance of PMMA interim restorations by adding various filler particles such as fibers [27, 28], NPs [29–33], and nanotubes [34–36]. The inclusion of inorganic nanofillers into PMMA changes the characteristics of the final product based on the size, shape, type, concentration, and filler to matrix interaction [33]. The present study aims to investigate the effect of the physical incorporation of TiO_2_ and ZrO_2_ NPs on the physical and mechanical properties of the PMMA-based provisional crown material, especially in terms of morphology, hardness, modulus, and hydrophilicity.

## 2. Materials and Methods

### 2.1. Materials

PMMA temporary resin acrylic (Bosworth, Trim Plus; Bosworth Company, USA), TiO_2_ (nanopowder, 21 nm, ≥99.5% trace metals basis; Sigma Aldrich, Germany), ZrO_2_ nanopowder (<100 nm particle size, Sigma Aldrich, China). The various test groups along with composition are given in Table 1.

### 2.2. Mixing of Fillers

All modified PMMA composites consisted of a liquid-to-powder ratio of 50/50 wt% (1 : 1 liquid-to-powder resin). TiO_2_ and ZrO_2_ NPs were added sequentially at 0.5, 1.5 and 3.0 wt% of each filler type, as indicated in Table 1. The required wt.% of filler for each group was dispersed into the powder resin by homogenizing it manually and mixing it by hand with a stainless steel spatula. The powder mixture with the filler was then mechanically mixed three times with an asymmetric double centrifuge at 1500 rpm, with two minutes pause in between.

### 2.3. Specimen Fabrication

A series of pristine (control) and modified PMMA composites (with 0.5, 1.5, and 3.0 wt%-TiO_2_/ZrO_2_) were prepared according to the scheme shown in Figure 1. Sixty bar (2 × 3 × 20 mm) and disc specimens (10 mm × 6 mm) were fabricated in six groups each (*n* = 10) for evaluation of their flexural strength and micro hardness. Silicone molds were developed to prepare the bar and disk specimens. The powder and liquid phases of the PMMA material (Bosworth Trim Plus, USA) were blended in a volume ratio of 1 : 1 and mixed with the NPs at low speed (1000 rpm for 60 seconds). The silicone molds were brought into contact with a glass slide, and the blended material was poured into them. After removing excess material, a glass slide was placed on the top of the mold until the material was fully polymerized. After complete polymerization, the specimens were stored at 37 °C for 1 hr before removing them from the molds. The specimens were allowed to cool for 30 minutes, removed from the molds, and polished with 600-1000-2400 grit SiC paper for 3 minutes. The specimens were then ultrasonicated with distilled water for 5 minutes to remove impurities and stored at 37 °C for 24 h.

### 2.4. Flexural Strength (Three-Point Bending)

For all specimens, a three-point bending test was performed on a universal testing machine (Instron Corp, Model:4202) using a crosshead speed of 0.5 mm/minute and a 100-kg load cell with a 3-point fixture with a span of 15 mm. The bars were oriented to allow high tensile force on the ground surface (bottom) and compression force on the top. The average heights and widths of the parts of the bars and the disc near the fracture point were measured with a micrometer (Model No. CD-4 C.S.; Mitutoyo Corp., Japan). The flexural strength (*σ*) and elastic modulus (*E*) are determined as follows:

(1) $$\begin{array}{c} \sigma =3\;PL/2\;WT2,\left(MPa\right) \end{array}$$

(2) $$\begin{array}{c} E=FL3/4WT3d,\left(MPa\right) \end{array}$$

where *P* is the maximum load (N) at fracture, *L* is the space amongst the two supports (fixed at 20 mm), *W* is the width of the bar (mm), and *T* is the height (mm). *F* is the applied force (N) and *d* is the deflection (mm) due to applied force F.

### 2.5. Microhardness Assessment

For microhardness testing, a Vickers microhardness indentation was applied to the disc specimens using a Vickers hardness tester (HMV-2 Shimadzu Corp, Tokyo, Japan). Three indentations were randomly placed on the surface of the specimen. The indentations were 0.5 mm apart and were loaded with 100 g for 15 s dwell period (ASTM C1327-03 standard). The average of the three readings for each specimen was determined as the individual Vickers hardness (V.H.).

### 2.6. Surface Roughness and Morphology

The surface roughness measurement was performed using a 3D non-contact optical microscope contour (GT-K 3D Bruker®). Specimens were measured using a 5× Michelson magnification objective, a field of view of 1.0 × 1.0 mm^2^, a Gaussian regression filter, a scan speed of 1×, and a threshold of 4× (vertical scan interferometry). The surface roughness was measured by following the same procedure previously published by our group [37]. In addition, the fractured structure morphology of all the specimens were investigated by scanning electron microscopy (JEOL, JSM-6610 LV, Tokyo, Japan) at 15 kv voltage and resolution from 100× to 500×.

### 2.7. Contact Angle Measurements

The water contact angle was measured at room temperature using a standard Ramé-Hart 250 goniometer and DROP image advanced software. The goniometer is equipped with a volume-controlled syringe above the substrate holder, a CCD camera that captures the droplet image, and DROPimage advanced software to process the data. The sessile drop technique was used, in which a 5 *μ*l drop of water was applied to a substrate, and the contact angle was measured within five seconds.

### 2.8. Statistical Analysis

A univariate two-way ANOVA was performed to analyze significant differences in F.S., EM, WCA, and VH between various test groups at *p* < 0.05 level of statistical significance.

## 3. Results and Discussion

### 3.1. Surface Roughness (Ra)

Figures 2(a)–2(d) show the surface roughness and topographic features of the pristine and TiO_2_/PMMA composites. Various mathematical models are used to measure the surface roughness based on the geometric topography. However, researchers mainly use average surface roughness (Ra) and root mean square roughness (Rq) to analyze surface roughness [17, 38–40]. The resulting values of the average surface roughness (Ra) of the control group and the TiO_2_ NPs reinforced group were recorded as 3.37 ± 1.45 *μ*m, 9.62 ± 0.84 *μ*m, 10.67 ± 1.36 *μ*m, and 11.59 ± 1.21 for the control, 0.5-TiO_2_, 1.5-TiO_2_, and 3-TiO_2_, respectively. Also, the root mean square roughness (Rq) was found to be 4.71 ± 0.86, 12.96 ± 0.69, 14.05 ± 1.37, and 14.93 ± 0.95 for the control, 0.5-TiO_2_, 1.5-TiO_2_, and 3-TiO_2_, respectively. Figures 3(a)–3(d) show the surface roughness and topographic properties of the control and ZrO_2_/Trim composites. The Ra values were 3.37±, 8.87±, 9.38 ±, and 10.52 ± for the control, 0.5-ZrO_2_, 1.5-ZrO_2_, and 3-ZrO_2_, respectively. Also, the Rq values were 4.71 ± 1.04, 12.18 ± 1.37, 12.71 ± 0.85, and 14.03 ± 1.54 for the control, 0.5-ZrO_2_, 1.5-ZrO_2_, and 3-ZrO_2_, respectively. In general, the surface of composites is influenced by many factors such as type and size of filler, shape, dispersion, type of resin matrix, degree of conversion, and bonding efficiency at the filler/matrix interface [41]. The results showed that the Ra of the modified PMMA composites marginally increased by increasing TiO_2_ and ZrO_2_ content. The steady increase in the surface roughness of the modified PMMA nanocomposites due to the incorporation of TiO_2_ and ZrO_2_ nanofillers could be due to the dispersion of these nanoparticles on the surface, resulting in an uneven surface [37, 42].

### 3.2. Flexural Strength and Vickers's Hardness

It is assumed that differences in filler content, type, size, and dispersion in the polymer matrix will influence the mechanical properties of the composite groups. Figures 4(a)–4(b) summarize the flexural strength (FS) and elastic modulus (EM) of the pristine and the different composite groups reinforced with TiO_2_ (0.5-TiO_2_, 1.5-TiO_2_, and 3-TiO_2_) and ZrO_2_ (0.5-ZrO_2_, 1.5-ZrO_2_, and 3.0-ZrO_2_). The FS and EM of pristine (control group) were measured to be 87.61 ± 3.21 MPa and 2865.32 ± 98 MPa, respectively. The inclusion of a small amount of TiO_2_ and ZrO_2_ (0.5 wt%) significantly increased the FS and EM values of the PMMA pristine interim restorative material. FS and EM values for 0.5-TiO_2_ were reported as 107.05 ± 5.11 MPa and 3434.70 ± 101 MPa, respectively. However, further increase in TiO_2_ content resulted in much lower FS values of 97.70 ± 4.51 MPa and 94.13 ± 3.98 for 1.5-TiO_2_ and 3.0-TiO_2_ respectively. Conversely, a gradual increase in EM was observed with increasing TiO_2_ filler content, with 3.0-TiO_2_ exhibiting the highest EM (3632.34 ± 89 MPa) compared to the other TiO_2_-containing groups. Similarly, 0.5-ZrO_2_ resulted in FS and EM values of 111.68 ± 4.35 MPa and 3445.52 ± 79 MPa, respectively. Increasing the ZrO_2_ filler content to 3.0 wt% resulted in a significant decrease in F.S., but EM was gradually increased with increasing ZrO_2_ content (from 3445.52 ± 79 for 0.5-ZrO_2_ to 3851.28 ± 112 for 3.0-ZrO_2_). Among the groups reinforced with ZrO_2_, 3.0-ZrO_2_ (due to the addition of 3 wt% nano-ZrO_2_) resulted in the highest EM (3851.28 ± 112).

When comparing the materials of the different test groups, the difference between FS and EM of the control group and the other groups can be explained on the basis of the type, size, and content of the fillers. In general, a good relationship between the mechanical strength and the filler's volume fraction is reported in the literature [43, 44]. Therefore, the composite groups with higher filler content are expected to exhibit higher mechanical strength than those with lower filler content. In the current study, lower FS was observed for 1.5-TiO_2_, 1.5-ZrO_2_, 3.0-TiO_2_, and 3.0-ZrO_2_, possibly due to the higher filler-to-matrix ratio and the presence of weak interaction between the filler and matrix materials. The increase in EM with increasing filler content could be attributed to increased stiffness [45]. These results are consistent with previous studies in which composites with high filler content exhibited high EM [46–48].

Figure 5 shows the Vickers hardness values for the pristine and composite groups. The pristine trim (control) resulted in a hardness value of 17.2 HV. The addition of TiO_2_ nanofiller resulted in a gradual increase in the micro hardness of composite groups from 22.65 HV for 0.5-TiO_2_ to 31.73 HV for 3.0-TiO_2_. A similar trend was observed for the composite groups modified with ZrO_2_, with microhardness values ranging from 21.82 HV for 0.5-ZrO_2_ to 27.84 HV for 3.0-ZrO_2_. In other words, 3.0-TiO_2_ showed the highest hardness values, followed by 3.0-ZrO_2_. The increase in microhardness of the modified PMMA nanocomposite groups could be related to the reduction in interparticle spacing As the particle loading in the polymer matrix increases, leading to an increase in surface resistance to indentation [49]. Shirkavand and Moslehifrad found in their study that the different ratio of PMMA reinforced with TiO_2_ increases the mechanical properties at a particular concentration and then decreased with an additional higher amount of TiO_2_ [22]. The required mechanical strengths of the composite materials may vary for intended applications. In some cases, high strength and hardness are required in the materials, while in others, flexibility, stiffness, and elasticity are the desired properties [48]. In conclusion, it can be assumed that by controlling the content of the above mentioned particles in PMMA nanocomposite groups, desired mechanical properties can be obtained.

### 3.3. Contact Angle

The contact angle values of all specimens were measured as an indicator of surface wettability and adhesion strength. It was found that increasing the surface roughness improved the wettability and decreased the contact angle value. A relationship exists between polymer surface roughness and liquid contact angles. A change in the surface roughness parameters of any material leads to a change in the contact angles or wettability of the material [50, 51].  Figure 6 shows the contact angle values of the PMMA pristine and nanocomposite specimens. Overall, the pristine specimen gave the highest contact angle (91.32 ± 4.21°). Among the TiO_2_ and ZrO_2_ composite groups, 0.5-ZrO_2_ gave the highest contact angle (83.10 ± 4.25°), followed by 0.5-TiO_2_ (81.06 ± 3.41°). Increasing the filler content (TiO_2_ and ZrO_2_) in the reinforced composites resulted in a gradual decrease in the contact angle. The lowest contact angle was obtained for 3.0-ZrO_2_ (66.30 ± 4.23), followed by 3.0-TiO_2_ (69.88 ± 3.55). The decrease in contact angle with increasing filler contact could be due to the increased surface roughness, as shown by the surface roughness measurement. It has already been shown that an increase in surface roughness improves the wettability and decreases the contact angle value [52].

Low contact angles indicate that the solid material is hydrophilic and the liquid spreads on the surface. In contrast, higher water contact corresponds to a hydrophobic solid and the liquid does not spread on the surface [53]. A water contact angle greater than 90° or slightly less than 90° corresponds to hydrophobic material, while a water contact angle of 51.05° ± 0.84° corresponds to a hydrophilic material. Complete wetting of material occurs when the contact angle is 0° [54] [55]. Therefore, based on the above findings, it can be inferred from the current study that the addition of more than 0.5 wt% TiO_2_ and ZrO_2_ nanofillers transforms the hydrophobic nature of the temporary crown material into a hydrophilic one.

### 3.4. SEM Analysis

Figures 7(a)–7(g) show the fractured cross-sectional microstructure of pristine, TiO_2_, and ZrO_2_ nanofilled composites. The analysis of SEM shows that the control group (Figure 7(a)) has a smooth microstructure compared to the nanofilled composites. However, with increasing concentration of the nanofillers TiO_2_ (Figures 7(b), 7(d), and 7(f)) and ZrO_2_ (Figures 7(c), 7(e), and 7(g)) (0.5 to 3.0 wt%), a rough microstructure with increasing micro cracks is observed. Composites with a lower concentration of nanofillers (0.5-TiO_2_ and 0.5-ZrO_2_) exhibited a corrugated fracture surface and showed warped and profound cracks on the surface. Moreover, no de-boned nanoparticles were observed on the surface, indicating that the nanoparticles were most likely enclosed by the polymer matrix chains, which indicated a good interaction between filler and polymer [37]. However, with increasing concentration (3.0-TiO_2_, 3.0-ZrO_2_), a ragged microstructure with deeper irregular cracks is obtained together with de-boned nanoparticles. The appearance of micro indentations and deep irregular cracks is induced by the pull-out of the resin-coated nanoparticles and indicates significant toughness. These morphological studies confirm the improvement of EM the nanoparticle-filled composites compared to pristine.

## 4. Conclusion

The physical incorporation of a small amount of TiO_2_ and ZrO_2_ (0.5 wt.%) as fillers into PMMA-based interim restorative material significantly improved the physical, mechanical, and morphological properties. The higher concentration of these fillers resulted in a decrease in FS. However, EM and surface hardness gradually increased with increasing filler content, with 3.0 wt.% ZrO_2_ exhibiting the highest EM (3851.28 MPa), followed by 3.0 wt.% TiO_2_ (3632.34 MPa). Moreover, a gradual increase in surface roughness was observed with increasing filler content. In addition, the water contact angle as a measure of wettability was significantly reduced from 91.32 ± 4.21° for the original PMMA to 66.30 ± 4.23° for 3.0 wt.% ZrO_2_ and 69.88 ± 3.55° for 3.0 wt.% TiO_2_. Thus, the higher content of TiO_2_ and ZrO_2_ increases toughness and stiffness on one hand and reduces hydrophobicity and flexibility of the composites on the other hand.

## Figures and Tables

**Figure 1:** Schematic diagram of the preparation of PMMA (TiO_2_/ZrO_2_) disk and bar specimens.

**Figure 2:** Surface roughness and topographic images of TiO_2_/Trim composites: (a) pristine PMMA, (b) 0.5-TiO_2_, (c) 1.5-TiO_2_, and (d) 3.0-TiO_2._

**Figure 3:** Surface roughness and topographic images of ZrO_2_/Trim composites: (a) pristine PMMA, (b) 0.5-ZrO_2_, (c) 1.5-ZrO_2_, and (d) 3.0-ZrO_2_.

**Figure 4:** Flexural strength (a) and elastic modulus (b) of the pristine and modified PMMA composite groups.

**Figure 5:** Vickers hardness values of the pristine and modified PMMA composite groups.

**Figure 6:** Water contact angle of the pristine and modified PMMA composite groups.

**Figure 7:** Scanning electron microscopy (SEM) images of fractured surface: (a) pristine PMMA, (b) 0.5-TiO2, (c) 1.5-TiO2, (d) 3.0-TiO2, (e) 0.5-ZrO2, (f) 1.5-ZrO2, and (g) 3.0-ZrO2.

**Table 1:** Material composition of the test groups.

S. no.	Group code	Description
1	Control	Pristine PMMA powder and liquid (1 : 1)
2	0.5-TiO_2_	PMMA powder + liquid (1 : 1) + 0.5 wt.TiO_2_
3	1.5-TiO_2_	PMMA powder + liquid (1 : 1) + 1.5 wt.TiO_2_
4	3.0-TiO_2_	PMMA powder + liquid (1 : 1) + 3.0 wt.TiO_2_
5	0.5-ZrO_2_	PMMA powder + liquid (1 : 1) + 0.5 wt.ZrO_2_
6	1.5-ZrO_2_	PMMA powder + liquid (1 : 1) + 1.5 wt.ZrO_2_
7	3.0-ZrO_2_	PMMA powder + liquid (1 : 1) + 3.0 wt.ZrO_2_

## Data Availability

The data used to support the findings of this study are included within the article.
